# Auricular Acupressure Therapy for Patients with Cancer with Sleep Disturbance: A Systematic Review and Meta-Analysis

**DOI:** 10.1155/2021/3996101

**Published:** 2021-10-14

**Authors:** Yunxia Wang, Jiayuan Zhang, Yuxia Jin, Qi Zhang

**Affiliations:** Chengdu University of Traditional Chinese Medicine, Chengdu, Sichuan Province, China

## Abstract

**Aim:**

We aim to provide available synthesized evidence of the efficacy and safety of auricular acupressure for cancer patients with sleep disturbance.

**Methods:**

Randomized controlled clinical trials (RCTs) were identified from PubMed, EMBASE, Web of Science, The Cochrane Library, PsycINFO, Chinese Biomedical Database, China National Knowledge Infrastructure, Chongqing VIP, and Wanfang Data, and the search date ranged from the inception of the databases to May 2021. Literature screening and data extraction were independently performed by three researchers. The Cochrane collaboration's tool for assessing the risk of bias was applied to evaluate the risk of bias of the RCTs included. The extracted data were analyzed using Rev-Man 5.4.1 software.

**Results:**

Nine trials involving 688 participants met the inclusion criteria and were included in the qualitative analysis; 6 trials involving 485 participants were included in the meta-analysis. Synthesized results showed that auricular acupressure had a significant effect on reducing the total Pittsburgh Sleep Quality Index (PSQI) score (MD = −3.88, 95% CI (−5.24, −2.53), *P* < 0.00001), and the scores of five PSQI components, sleep latency (MD = −0.53, 95% CI (−0.73, −0.32), *P* < 0.00001), subjective sleep quality (MD = −0.79, 95% CI (−1.05, −0.53), *P* < 0.00001), sleep duration (MD = −0.50, 95% CI (−0.69, −0.31), *P* < 0.0001), daytime dysfunction (MD = −0.53, 95% CI (−0.77, −0.29), *P* < 0.0001), and sleep disturbances (MD = −0.54, 95% CI (−0.60, −0.49), *P* < 0.00001), were also obviously decreased after the intervention of auricular acupressure. Shenmen and heart were the most commonly selected auricular acupoints, the main intervention durations ranged from 10 to 42 days, and the pressing times of auricular acupoints were 1–6 times a day, 1–5 min each time. One trial reported slight and transient pain caused by auricular acupressure, while the remaining 8 trials did not report obvious side effects.

**Conclusion:**

Auricular acupressure can significantly improve the sleep quality of cancer patients with sleep disturbance, with no obvious side effects. Rigorously designed clinical trials are necessary for the further support of the clinical application.

## 1. Introduction 

Insomnia is highly prevalent in cancer patients; on the basis of the relevant researches, sleep disturbance is one of the most common complications in cancer patients, with a prevalence of 19%–75% [1–3], which seriously influences the mental and physical health of cancer patients [4]. It has been reported that the prevalence of sleep disturbance in cancer patients is greater than that in the general population [4], especially in patients with lung cancer and breast cancer [5]. Sleep disturbance can be seen in the process of diagnosis and anticancer treatment and can persist for a long time in cancer survivors [5,6]. There are many factors that can cause sleep disturbance in cancer patients, such as the symptoms of cancer, anticancer treatment, and psychological causes [7, 8]. Due to the various causes, the manifestations of sleep disturbance in cancer patients are also different [8–10]. A study [11] of 426 cancer patients who received chemotherapy showed that 73.2% reported difficulty in falling asleep, 56% reported waking up in the middle of the night, and 65% reported waking up earlier than expected in the morning. In addition, sleep disturbance often occurs in the form of cancer symptom clusters in cancer patients; the most common symptom clusters [12, 13] of cancer patients are gastrointestinal symptom cluster which is composed of nausea, vomiting, and loss of appetite, as same as psychoneurological symptom cluster with pain, fatigue, and sleep disturbance or fatigue, depression, and sleep disturbance. Symptoms in the same symptom cluster interact with each other, and the treatment for a single symptom may be ineffective. Sleep disturbance can lead to a decreased quality of life in cancer patients and may cause and worsen the symptoms such as fatigue, depression, pain, and infections [2, 4, 7, 14, 15] and even reduce the survival rate of cancer patients [16]. Despite the great prevalence of sleep disturbance in cancer patients, it has been reported that the symptoms of sleep disturbance were often neglected and not properly managed [14, 17, 18]. The sleep disturbance in cancer patients is mainly treated with hypnotic drugs, but hypnotic drugs are only recommended for short-term use, and long-term use of them may cause drug tolerance and drug dependence [19] and can increase the risk of daytime dysfunction, cognitive dysfunction, fall, and other adverse events [5, 7]. Pharmacotherapy for cancer patients with sleep disturbance also has to take into account the concomitant interactions with current anticancer medication [19]. In addition, in an epidemiological trial of 5000 sleep medication users, 80.3% of them prefer nonpharmacological therapies; however, only 9.6% of them have actually received nonpharmacological treatment [20].

Since sleep disturbance in cancer patients is common and chronic, it is necessary to explore nonpharmacological therapy. Recently, the therapeutic effect of several nonpharmacological therapies on improving sleep disturbance in cancer patients has been reported, including cognitive intervention [21], aerobic exercise [22], and somatic acupoints stimulation [23]. The positive effect of auricular acupressure on improving sleep disturbance has been confirmed by several trials, which has the advantages of simple operation and few side effects [24–26]. Auricular acupoints are considered to be the projection of the whole human body, and auricular acupressure is to stick the vaccaria seeds or magnetic beads on the auricular acupoints and adjust the function of the whole body by pressing and stimulating the auricular acupoints [27, 28]. This study aims to assess the therapeutic effect of auricular acupressure for cancer patients with sleep disturbance and provide available evidence for selecting auricular acupressure as a nonpharmacological therapy for cancer patients with sleep disturbance.

## 2. Materials and Methods

### 2.1. Registration

The protocol of this systematic review has been registered in PROSPERO (Registration Number: CRD42021209436).

### 2.2. Inclusion Criteria

#### 2.2.1. Types of Trials

The randomized controlled clinical trials (RCTs) will be included.

#### 2.2.2. Types of Patients

Cancer patients over 18 years old with an accurate diagnosis of sleep disturbance are included, and there is no restriction on the type or stage of cancer.

#### 2.2.3. Types of Interventions

(1) The intervention of included trials was limited to only auricular acupressure, and the pressing materials can be vaccaria seeds, magnetic beads, and so on. Nonpressing treatments such as acupuncture or laser at the auricular acupoints will be excluded, and other types of acupressure, massage, acupuncture will be excluded. (2) The treatment of the control group includes routine care, sham acupressure, pharmacotherapy, or no intervention.

#### 2.2.4. Types of Outcomes

The main outcomes are as follows: (1) Subjective measurement: standardized changes in Pittsburgh Sleep Quality Index (PSQI) or other scales that are widely applied for measuring sleep quality. A specific scale for measuring sleep quality is required, and an option for measuring sleep quality contained in a certain scale will be excluded. (2) Objective measurement: polysomnography (PSG), actigraphy, and so on.

The secondary outcomes are as follows: (1) adverse events, (2) compliance, and (3) follow-up.

### 2.3. Search Strategy

Literature searching covered both English and Chinese electronic databases, including PubMed, Web of Science, EMBASE, The Cochrane Library, PsycINFO, Chinese Biomedical Database, China National Knowledge Infrastructure, Wanfang Data, and Chongqing VIP. Medical subject headings combined with text word searching were performed, and the search date ranged from the inception of databases to May 2021.

### 2.4. Data Collection and Analysis

#### 2.4.1. Selection of Trials and Data Extraction

Trials selection was performed independently by three researchers (Yunxia Wang, Yuxia Jin, and Jiayuan Zhang), and the unified scale and cross-checking were conducted. We contacted the author to obtain the necessary data when the required information was incomplete. The decision of including a controversial trial was made by a fourth researcher (Qi Zhang). The entire process was performed in the Preferred Reporting Items for Systematic Reviews and Meta-Analyses (PRISMA) flow diagram.

#### 2.4.2. Assessment of Risk of Bias

The Cochrane collaboration's tool for assessing the risk of bias was applied to assess the risk of bias of the trials included, which is categorized as “low risk” of bias, “unclear risk” of bias, or “high risk” of bias.

#### 2.4.3. Measures of Treatment Effect

The extracted data were analyzed by the Rev-Man 5.4.1 software provided by the Cochrane collaboration, for dichotomous variable, 95% confidence intervals (95% CI), and risk ratio (RR) was reported; meanwhile, for a continuous variable, 95% confidence intervals and mean difference (MD) were reported.

#### 2.4.4. Assessment of Heterogeneity and Data Synthesis

*Q*-statistic and *I* [2] statistic were performed to evaluate statistical heterogeneity. The data were assessed by the fixed-effects model when there was no significant heterogeneity (*P* > 0.10, *I*^2^ < 50%). Otherwise, the data was assessed by the random-effects model (*P* < 0.10, *I*^2^ > 50%).

#### 2.4.5. Assessment of Reporting Bias

When the included trials were more than 10, publication bias was assessed by a funnel plot.

#### 2.4.6. Subgroup Analysis and Sensitivity Analysis

Subgroup analysis (grouped by age, cancer type, anticancer treatment, and interventions) and sensitivity analysis were conducted when there was significant heterogeneity.

## 3. Results

A total of 132 literature studies were identified, among which 52 duplicate literature studies were removed, 46 irrelevant literature studies were excluded after reading the title and abstract, and 25 literature studies were excluded after reading the full text. Finally, 9 trials [29–37] met the inclusion criteria and were included in qualitative analysis, 6 trials were included in the meta-analysis, and the screening results are shown in Figure 1.

### 3.1. Characteristics of the Included Trials

Among the 9 trials that finally met the inclusion criteria for qualitative analysis, the publication time was from 2014 to 2019, 7 trials were from China, 2 trials were from Korea and Britain, involving 688 participants, 3 trials were published in English, and 6 trials were published in Chinese. The cancer types of included trials were 1 primary liver cancer, 1 lung cancer, 2 breast cancer, 1 ovarian cancer, 3 recruited patients with different cancer types, and 1 not explicitly reporting the cancer type. Cancer staging covers I–IV. Anticancer treatments included surgery, radiotherapy, and chemotherapy. Patients in the intervention group were treated with auricular acupressure alone, while the control group was treated with routine nursing (*n* = 8), sham acupuncture (*n* = 1), and no treatment (*n* = 1). The intervention time ranged from 10 to 42 days, and the pressing times of auricular acupoints were 1–6 times a day, 1–5 min each time. The subjective sleep quality measurement was 6 trials with PSQI, 1 trial with PSQI and Self-Rating Scale of Sleep, and 2 trials with Athens Insomnia Scale (AIS). As for the objective measurement, only 1 trial reported the data of fit bit tracker for 24 hours and the sleep quality-related blood inflammatory indicators values including IL-6, TNF-*α*, cortisol, and CRP levels. The total number of patients included in the meta-analysis was 485, including the intervention group (241 participants) and the control group (244 participants). The general characteristics of the included trials are shown in Table 1.

### 3.2. Risk of Bias of the Included Trials and Methodological Quality

The risk of bias assessment for the included trials is shown in Figure 2. In the aspect of random sequence generation, 5 trials used a table of random numbers and 1 trial conducted 1 : 1 allocation ratio by lot. As for allocation concealment, only 1 trial mentioned that the randomized personnel had no contact with the participants. In the aspect of blindness, 1 trial was blind to the subjects applying sham auricular acupressure, 1 trial was blind to the results, and the other 4 trials did not mention blindness; however, the control group of these trials adopted routine nursing and no treatment, due to the particularity of auricular acupuncture treatment, and it can be seen that the blindness to the subjects of these 5 trials has not been implemented. Drop-out of participants occurred in 3 trials, the number of drop-out participants was small and was similar between the intervention group and the control group, and the causes of drop-out were all reported in detail. No research protocol was found for 6 trials, and 1 trial reported all prespecified outcomes.

### 3.3. Auricular Acupoints Selection for Cancer Patients with Sleep Disturbance

Among the 9 trials included in the qualitative analysis, regarding the standards of auricular acupoints selection and location for the intervention group, 1 trial adopted the new Chinese national standard nomenclature and locations of auricular acupuncture points (GB/T13734-2008) [38], and 1 trial adopted the methods of referring to acupuncture/acupressure textbooks and consulting acupuncturists, while the standards of auricular acupuncture points were not reported in the other 7 included trials. Unilateral auricular acupressure was conducted in 5 trials, and the adhesive tape attached to ear was replaced to the other ear in 1–6 days. Binaural auricular acupressure was performed in 4 trials, and the adhesive tape attached to ear was replaced in 2–7 days. 3–7 auricular acupoints were mainly selected in the included 9 trials, and the most commonly selected auricular acupoints were Shenmen and the heart (9 trials), followed by subcortical (7 trials), then endocrine, occipital, and sympathetic nerve (3 trials), and liver, spleen, and kidney (2 trials). The intervention durations were 10–14 days (3 trials), 28–30 days (3 trials), and 35–42 days (3 trials), respectively. As for the number of pressing times, 2 trials were once a day (1 min each time), 4 trials were 3–5 times a day (3–5 min each time, 1 trial was 20–30 press each time), 2 trials were 5–6 times a day (1-2 min and 500–600 press each time, respectively), 1 trial did not report the number of pressing times, and only one mentioned pressing every day (2-3 min each time).

### 3.4. Scores of Sleep Quality Index

In the 9 trials included qualitatively, 1 trial [31] showed no statistically significant difference in the AIS score between the intervention group and the control group after the intervention of auricular acupressure, and the other 8 trials reported that the PSQI score (*n* = 7) and AIS score (*n* = 1) in the intervention group were significantly lower than those in the control group and the sleep quality was significantly improved after the intervention, while there was no significant difference in PSQI score between the two groups before the intervention of auricular acupressure. Meta-analysis was carried out on the total scores of PSQI in 6 trials included, synthesized results showed that auricular acupressure had a significant effect on reducing the total PSQI score (MD = −3.88, 95% CI (−5.24, −2.53), *P* < 0.00001), and the results are shown in Figure 3.

Due to the high heterogeneity (*I*^2^ = 91%, *P* < 0.00001), sensitivity analysis and subgroup analysis were performed. The 6 included trials were removed one by one in sensitivity analysis, and the heterogeneity of the synthesized results did not decrease significantly. After deleting the study by Kuo et al. with the greatest intervention effect and the study by Wei and Zhang with the smallest intervention effect, the heterogeneity of the remaining 4 trials decreased significantly (*I*^2^ = 0%, *P*=0.59), and the synthesized results were (MD = −3.46, 95% CI (−4.05, −2.87), *P* < 0.00001), which still showed that the PSQI score of the intervention group was significantly lower than the control group (*P* < 0.00001), indicating that the synthesized results were stable. Subgroup analysis was conducted according to the intervention duration and sample size, the heterogeneity decreased slightly, and no significant differences were found between subgroups.

Among the 6 trials applying PSQI, 3 trials reported the scores of five PSQI components, which were also analyzed by meta-analysis. The synthesized results showed that sleep latency, subjective sleep quality, sleep duration, daytime dysfunction, and sleep disturbances were obviously improved after the intervention of auricular acupressure, as shown in Figure 4.

### 3.5. Objective Measurement of Sleep Quality

Only 1 trial [36] reported the objective measurement of sleep quality, and the results of fit bit tracker device data showed that no significant differences were found in total sleep time, sleep latency, sleep efficiency, or number of times awakened during sleep between the intervention group and the control group after intervention; meanwhile, significant differences in blood tests for IL-6 level and TNF-*α* level between the two groups were found, while no significant differences were found in cortisol level and CRP level.

### 3.6. Side Effects

Trial [34] reported that 2 participants mentioned the slight pain and discomfort caused by auricular acupressure, while the remaining 8 trials [29, 33, 35–37] did not report obvious side effects.

### 3.7. Compliance and Follow-Up

Among the 9 trials included qualitatively, 36 participants dropped out in 1 trial, including 26 in the intervention group and 10 in the control group. The drop-outs related to intervention treatment were that 11 participants dropped out due to the foreign body sensation of auricular acupressure and 1 participant due to the inability to conduct auricular acupressure. The other drop-outs are due to death (*n* = 5), critical illness (*n* = 3), hospital transfer (*n* = 2), taking sleeping pills(*n* = 6), loss of contact (*n* = 4), cancer-related symptoms (*n* = 3), and refusal of results measurement (*n* = 1). Drop-outs were reported in the 3 trials included in the meta-analysis. In Lei [33], 2 participants dropped out in the intervention group, 1 voluntarily quit, and 1 quit after hospital transfer. In Kuo et al. [37], 3 participants dropped out in the intervention group, because of the inability to conduct auricular acupressure, while in the control group, 4 participants dropped out due to hospital transfer. In Yoon and Park [36], 1 participant in the intervention group voluntarily quit, the remaining 2 participants and 2 participants in the control group dropped out due to refusal of results measurement. None of the included trials conducted a follow-up study; thus, the long-term efficacy of auricular acupressure is unknown.

## 4. Discussion

To our knowledge, this is the first systematic review and meta-analysis on the therapeutic effect of auricular acupressure for cancer patients with sleep disturbance, which preliminarily confirmed the effectiveness and safety of auricular acupressure for cancer patients with sleep disturbance. In order to accurately evaluate the effect of auricular acupressure in cancer patients with sleep disturbance, the intervention of the included trials was limited to auricular acupressure, and the cancer patients were definitely diagnosed with sleep disturbance according to the relevant diagnostic criteria.The methodological lacks of included trials are mainly in the allocation concealment, implementation of blind method, and selective outcome reporting. Most of them can be improved by the rigorous design of the study according to the relevant guidelines. Among them, due to the particularity of auricular acupressure, there are certain restrictions on blinding of participants. The control group of included trials mostly adopts routine nursing, only 1 trial [36] adopts sham acupressure, it selected the acupoints of auricle as sham auricular acupoints, thus implemented blinding of participants and reducing the placebo effect, and it can be used as a reference for the future researches.

In the included trials, the shortest intervention duration of 10 days showed a significant effect on improving sleep quality. The synthesized results showed that auricular acupressure can significantly reduce the total PSQI score and the scores of five PSQI components, and another trial [39] also reported decreased scores in 5 PSQI components after the intervention of auricular acupressure. The high heterogeneity of the synthesized results may be caused by the inconsistency of cancer types, intervention time, sample size, and so on. Compared with nonpharmacotherapy, hypnotic drugs are only recommended for short-term use due to the side effects, and they can only improve sleep induction, but not enough to improve sleep quality and prevent daytime dysfunction [14]. Melatonin is another medication commonly used for sleep disturbance; however, it has been reported that melatonin is ineffective for secondary sleep disturbance and has the side effects of dry mouth and constipation [5, 40]. It has already been reported in several studies that auricular acupressure has the therapeutic effects of improving nausea, vomiting [41], constipation [42], pain [43, 44], fatigue [28], and life quality [45] in cancer patients, and a randomized controlled study [46] reported significant clinical improvements in the symptom clusters of pain, fatigue, and sleep disturbance in cancer patients after 4 weeks of auricular acupressure. A meta-analysis [47] reported that, compared with estazolam, auricular acupressure could significantly increase the response rate (reduction of PSQI global score by 25% and more) in patients with maintenance hemodialysis (RR = 1.21, 95% CI: 1.04 to 1.40). Another meta-analysis [24] for patients with hypertension showed that a significant improvement of sleep quality was found in the auricular acupressure plus hypnotic medication group in comparison with the hypnotic medication group (MD = −0.71, 95% CI −3.86 to −2.43). One meta-analysis [26] for primary insomnia also reported that the PSQI score was lower in the auricular acupressure group than that in the medication group after the intervention (MD = −3.62, 95% CI −4.59 to −2.65).

At present, the researches on the mechanism of auricular acupressure for sleep disturbance are still insufficient. One of the included trials [36] suggests that auricular acupressure may improve sleep disturbance by reducing the levels of inflammatory cytokines in the blood and improving the inflammatory state after chemotherapy. Another study [48] indicates that auricular acupressure may improve sleep quality by increasing heart rate variability, as well as lowering blood pressure and heart rate. One study [49] reported that microcurrent stimulation at Shenmen acupoint could promote EEG changes related to sleepiness and positive mood. Another study [50] found that acupuncture can significantly increase endogenous melatonin secretion at night, which may be one of the mechanisms for improving sleep quality. Future researches should focus more on the objective measurements of sleep quality, so as to further reveal the possible mechanism of auricular acupressure for improving sleep disturbance.

Another problem found in this study is that the standards of auricular acupoint selection were not uniform. Only one included study [33] explicitly reported the standard of auricular acupoints selection and location, while it has been reported [26] that the inconsistent standard of auricular acupoints was one of the reasons affecting the efficacy of auricular acupressure. Compared with acupuncture, auricular acupressure is easy to operate and reduces the side effects of pain, bleeding, and infection, the slight pain caused by auricular acupressure has been reported to be tolerated after the treatment continued for one week [35], and the presses on alternate ears and hypoallergenic tape can be applied to further alleviate them. In terms of compliance, the main causes of drop-out due to the intervention of auricular acupressure are foreign body sensation of the ear and inability to press auricular acupoints; in this case, patiently educating and guiding participants and their caregivers about how to precisely locate and press auricular acupoints before starting treatment can play a certain role, and when the adhesive tape attached to ear falls off outside the hospital, participants and their caregivers can replace and supplement the adhesive tape to continue the treatment. At last, a follow-up study after intervention should be carried out to clarify the long-term efficacy of auricular acupressure, one study [46] reported that auricular acupressure could improve the sleep quality of cancer patients for one month after the intervention, and another study [51] showed that the sleep quality improvement effect lasted for six months in elderly people.

The main limitations are as follows: firstly, only Chinese and English databases have been searched, the studies reported in other languages may be missed. In addition, due to the limited study design of included trials, the evidence of synthesized results is inadequate.

## 5. Conclusion

Auricular acupressure can significantly improve sleep quality of cancer patients with sleep disturbance, with no obvious side effects. More high-quality, multicenter, and large sample size clinical trials are necessary for the further support of clinical application.

## Figures and Tables

**Figure 1:** Flow of literature screening.

**Figure 2:** Risk of bias of the included trials.

**Figure 3:** Forest plot of PSQI scores.

**Figure 4:** Forest plot of scores of five PSQI components.

**Table 1:** Characteristics of included trials.

Author (year)	Country	Sample sizes (M/F)	Mean age (I/C)	Diagnosis	Cancer stage	Diagnostic criteria of insomnia	Criteria of auricular acupoints	Anticancer treatment	Intervention material	Control	Acupoint selection	Course of treatment	Outcome measures	Adverse effects	Drop-out (I/C)	Follow-up
Lei (2019)	China	96 (60/36)	51.49 ± 8.40/52.49 ± 7.09	Primary liver cancer	I–III	PSQI > 7	GB/T13734-2008	Surgery or other therapies	Vaccaria seeds	Routine care	Shenmen, subcortex, heart, sympathetic nerve, endocrine, liver, and spleen	3–5 min/time, 3 times/d, 28 d	PSQI and SRSS	None	I2/C0	Not reported
Lu (2017)^*∗*^	China	60 (42/18)	Not reported	Lung cancer	Not reported	Not reported	Not reported	Radiotherapy	Vaccaria seeds	Routine care	Heart, Shenmen, anterior lobe, occiput, and subcortex	10 press/time, 5-6 times/d, 30 d	AIS	None	None	Not reported
Kuo (2018)	China	47	51.5 ± 13.23/54.7 ± 14.56	Ovarian cancer	I–IV	PSQI > 5	Not reported	Chemotherapy	Vaccaria seeds	Routine care	Shenmen, heart, subcortex, and endocrine	3 min/time, 3 times/d, 6 w	PSQI	None	I3/C4	Not reported
Yoon (2019)	Korea	46	45.05 ± 8.33/44.57 ± 8.34	Breast cancer	I–III	ISI ≥ 8	Not reported	Chemotherapy	Vaccaria seeds	Placebo auricular pressure (helix control points)	Shenmen, heart, anterior lobe, and occiput	1 min/time, once/d, 6 d/w, 6 w	PSQI, IL-6, TNF-*α*, cortisol, C-reactive protein, and fit bit tracker device	None	I3/C2	Not reported
Lin (2018)	China	60	36.41 ± 9.13/37.27 ± 10.21	Breast cancer	II	The Chinese Classification and the Diagnose Criterion of Mental Disorder	Not reported	Chemotherapy	Vaccaria seeds	Routine care	Shenmen, heart, kidney, subcortex, and sympathetic nerve	3–5 min/time, 3–5 times/d, 11 d	PSQI	None	None	Not reported
Hughes (2015)^*∗*^	Britain	6 (2/4)	52.25 ± 12.31/54.00 ± 2.83	Breast cancer 4 and colorectal cancer 2	Not reported	PSQI ≥ 5	Acupuncture/acupressure textbooks; consult an acupuncturist	Chemotherapy or radiotherapy	Vaccaria seeds	No treatment	Bilateral Shenmen, any two from insomnia 1, insomnia 2, heart, liver, kidney, and subcortex	1 min/time, once/d, 35 d	PSQI	Slight, transient pain of the ear	None	Not reported
Wei (2019)	China	148 (80/68)	59.28 ± 9.41/59.14 ± 9.23	Lung cancer 30, intestinal cancer 18, gastric cancer 8, breast cancer 8, and pancreatic cancer 10	Not reported	Guidelines for diagnosis and treatment of insomnia in Chinese adults	Not reported	Not reported	Vaccaria seeds	Routine care	Shenmen, heart, endocrine, and spleen	1-2 min/time, 6 times/d, 14 d	PSQI	None	None	Not reported
Song (2014)	China	100	Not reported	Gastric cancer 40, lung cancer 40, liver cancer 12, and gallbladder cancer 8	Not reported	PSQI	Not reported	Chemotherapy	Vaccaria seeds	Routine care	Subcortex, heart, sympathetic nerve, Shenmen, sympathetic nerve, ear apex, and brain stem, combined with liver, gallbladder, lung, and stomach	2-3 min/time, 10 d	PSQI	None	None	Not reported
Fan (2015)^*∗*^	China	125	60.0 ± 14.4/63.2 ± 13.5	Not reported	Not reported	CAIS-8 ≥ 8	Not reported	Chemotherapy, CCRT, or other therapies	Magnetic beads	Routine care	Shenmen, heart, occiput, and subcortex	20–30 press /time, 3 times/d, 28 d	AIS	None	I26/C10	Not reported

^*∗*^Qualitative inclusion; M/F: male/female; I/C: invention/control; AIS: Athens Insomnia Scale; ISI: Insomnia Severity Index; SRSS: Self-Rating Scale of Sleep; PSQI: Pittsburgh Sleep Quality Index.

## Data Availability

No data were used to support this study.

## Abbreviations

RCTs: Randomized controlled clinical trials
PSQI: Pittsburgh Sleep Quality Index
PRISMA: Preferred Reporting Items for Systematic Reviews and Meta-Analyses
95% CI: 95% confidence interval
RR: Risk ratio
MD: Mean difference
AIS: Athens Insomnia Scale.
